# Clinical Intervention Effect of a Predictive Model Constructed Based on Risk Factors for Falls in Elderly Patients during Hospitalization

**DOI:** 10.1155/2022/4983254

**Published:** 2022-09-23

**Authors:** Lizhi Wu, Lin Zhou

**Affiliations:** ^1^Pharmacy Intravenous Admixture Services, Wenling First People's Hospital, Wenling, Zhejiang 317500, China; ^2^Department of Integrated Traditional Chinese and Western Medicine, Department of Geriatrics, Wenling First People's Hospital, Wenling, Zhejiang 317500, China

## Abstract

Falls in elderly patients are an important cause of fractures, functional impairment, and mortality. In this paper, a questionnaire was used to collect information on fall history, balance function and sensory function from patients over 65 years of age. In the analysis, the presence or absence of falls was used as a factor, and a corresponding prediction model was constructed using methods such as univariate analysis and regression analysis. This survey found that in the past year, 60% of the patients had fallen, 16.67% had one fall, 33.33% had two falls, and 50% had three or more falls; model specificity is 61.54%, the sensitivity is 71.43%, and the misjudgment is 38.46%. The model has good specificity and sensitivity and a small misjudgment rate; so, the model is more reasonable. This paper selects several sensitivity indices that have a certain impact on the risk of falling and makes a satisfactory forecast, which can provide a theoretical basis for the prevention of the risk of falls in elderly patients during hospitalization.

## 1. Introduction

Since the 1950s, researches on falls of the elderly at home and abroad have been carried out in foreign countries, but due to their own reasons, there are a lot of literature in China [1, 2]. The mechanism of fall includes the central nervous system, musculoskeletal system, and proprioception. At present, there are many studies on the prevention and treatment of falls and injuries [3]. For example, the elderly are prone to fractures after a fall, among which hip fractures are the most common. Therefore, researchers in this area have developed protective measures in this area and have achieved good follow-up results [4]. Second, external factors have a certain impact on falls, such as the environment. Therefore, some scholars start with how to reduce the risk of falling from the external environment, such as scientific planning of the home environment and the production of nonslip shoes. In terms of rehabilitation medicine, it is mainly necessary to start from the cause and take corresponding measures to reduce the risk of falling. Numerous interventional studies have shown that exercise can effectively reduce the risk of falls.

In the past literature, most researchers used different assessment methods to assess the risk of falling [5–7], for example, DGI assessment scale, Berg balance scale, etc., to evaluate the balance of the individual, and then to further reflect the risk of falling. The higher the score, the better the balance and the lower the risk of falling. In addition, TUGT is a standing walking test at a designated time to measure the balance state of the subjects. It is better to take less than 20 seconds, and there is a risk of falling if more than 30 seconds. There are subjective factors in the above evaluation methods, and there is a lack of objective, reasonable, and comprehensive evaluation methods [8].

Recent years, there have been some nonlinear research methods such as local dynamic stabilization, which can reflect the changes of the gait of the elderly over time [9]. They can also track the elderly and people who have not fallen. Quandt et al. report that the Lyapunov index (LEE) derived from the upper body acceleration of the upper body shows that the local dynamic stability of the medial outer edge (ML) changes between different age groups [10]. It was found that its local stability decreased with aging. Similar findings were reported by Buz et al. The LEE was derived from the longitudinal movement time-course data of the lower extremities, and the LEE values were higher than in elderly patients. LEE shows age-related changes in gait control; so, LEE also has the potential to predict fall risk. Bisi et al. combined the timing of linear body acceleration in various directions to analyze and compare the LEE of children and adolescents. Children have higher levels of LEE, and it is certain that children's pace stability will be reduced.

Kukidome et al. reported that 20% of older adults at risk of falling at baseline improved after falling; meaning, their odds of falling increased as the risk of the problem increased reduce [11]. The Turkeli S system designed a suitable algorithm and a wearable electronic device for the elderly, a Tesodev-type drop detector [12]. Yanping et al. applied back-propagation multilevel neural networks to predict the risk of falling from a physiological perspective [13]. Peng developed a hazard and detection system and applied it to the homes of 19 elderly people. The system consists of Doppler radar, Microsoft Kinect, and 2 cameras [14]. By collecting data, comparing it with sensor data, and calculating and developing, it helps the elderly to maintain a normal life. At present, there are many monitoring instruments and means about falls of the elderly in my country, but the relevant literature on preventing falls is rare. Fall risk is a combination of multiple systems, but, whatever the reason, identifying specific factors that help increase risk can help adjust intervention strategies or change the situation to reduce the chance of falls.

At present, the relevant data on the risk of falls in elderly patients are relatively abundant, but from the point of view of biomechanics, there is no relevant data for reference. In this paper, various measurement methods are used to collect different viewing angle indices, a relatively complete analysis of the gait characteristics of the elderly and the correlation between various parameters is carried out, and a prediction model is established using appropriate statistical methods, so as to provide a better understanding of the elderly. The in-depth study of the biological mechanism of patient falls has laid the foundation.

## 2. Research Objects and Methods

### 2.1. Research Object

20 elderly patients, including 12 women and 8 men (65-75), were included in this study, and their height, weight, and BMI were measured [15]. Recruitment conditions have the ability to actively participate in the trial and have a clear willingness to know. Before the test, the operator explained the test process and operation points and completed the relevant operations. The following is the basic information of the subjects, see Table 1.

### 2.2. Research Methods

#### 2.2.1. Questionnaire Survey Method

This paper adopts The Tinetti-style “balanced volume” developed by Tinetti et al. which serves as a general method for assessing fall risk in the elderly. The test is divided into gait and balance. The balance test includes 10 items such as standing balance, sitting balance, standing balance, turn-standing balance, and jogging response, all of which are 16 items, of which 8 items include starting, striding, swinging foot height, symmetry, and continuous width, a total of 12 a [16]. A score lower than 24 points indicates a risk of falling, walking path, and trunk sway, with a score of 0.70 and a specificity of 0.53.

#### 2.2.2. Experimental Method

*(1) Visual Test*. In order to reduce the measurement error and ensure the accuracy and reliability of the data, a vision meter based on a vision meter is used [17]. In the experiment, the distance between the experimental subject and the target was 5 meters, the left eye and the right eye were tested once, one side was blocked, and then the final vision was statistically processed by the binocular average.

*(2) Proprioceptive Test*. This paper adopts the Biodex isokinetic muscle strength measurement device measured the upper limb flexion of the subjects. During this period, in order to avoid the influence of vision and hearing, it needs to be performed under silent conditions.

Active position sense was as follows: the starting position of the isokinetic muscle force meter is 90 degrees of knee flexion, the end position is to extend the knee joint 45 degrees, and the movement is carried out at a rate of 5 degrees/s. In the test, participants started from the starting point, and the lower limbs first performed knee flexion activities until the posture was completed, held for 10 seconds, and then returned to the starting point. When you reach the starting point, press the button to complete your trial. The above experiment was repeated 3 times and averaged. The effect of active positioning is evaluated according to the difference between actual positioning and set positioning. During the test, the subject should concentrate and not be distracted.

Passive position sense was as follows: the device settings are the same as above. In the test procedure, when the subject is in a passive state, press the button to complete the test.

*(3) Static Balance Test*. This test uses the German Zeeblis capacitive foot pressure tester. In the test, when the subject is standing, the heels are separated by 3-4 cm, the toes are 25-30 degrees, and the hands are naturally placed on both sides. While sitting, the eyes are looking straight ahead; when standing on one foot, the experimenter is in the center of the test platform, one foot is off the ground, the knee is bent, and the eyes are looking straight ahead. When the subjects were standing upright, their eyes looked straight at the wall, their eyes looked straight at a fixed object on the wall, and then they put their hands on their side; when they closed their eyes, they were tested. The subject stood on the test platform with his hands by his side, eyes closed, and his face facing forward.

Note that the test is divided into bipedal and monopedic, and the subject's body is measured without external force. The test period of each method is 10 seconds, the test data is recorded in real time, and the data is counted.

*(4) Stability Limit Test*. This part of the test uses the Tecnobody balance test and training system. Before the test, the subject stood in the middle of the test platform, that is, on both sides of Al, with the heels of both feet together, the second toes of both feet corresponding to A2 and A8, respectively, and their hands on their chests. During the test, subjects were required to move as far as possible in the directions of Al, A3, A5, and A7. During the exercise, flexion of the hips, knees, and heels were not allowed. Observe the angle of inclination in 4 directions, and the smaller the angle, the higher the risk of falling.

*(5) Gait Test*. The study subjects wore experimental clothing, wearing their usual shoes, and no jewelry, while the women had their hair tied up. Before the test, the experimenter will guide the subjects to make adjustments on other treadmills to avoid results that do not match the treadmill. During the trial, walking trials were performed according to the participants' walking rate, with a staff member behind them to provide safety.

## 3. Research Result

The analysis discusses data comparisons between fallen and nonfalling patients, occurrence of falls, and screening predictors.

### 3.1. Occurrence of Fall Events

The subjects of the study were fall accidents. After the trial was completed, 15 older adults were followed. The study found no statistically significant difference in the subjects' falls before and after the trial. Therefore, before the experiment, we will still select the fall situation as the follow-up analysis. According to statistics, in the past year, 60% of the patients had fallen, 16.67% had one fall, 33.33% had two falls, and 50% had three or more falls, see Figure 1.

In the past year, 12 women had a 60% chance of falling; 8 men had a 40% chance of falling. Statistical analysis based on underlying details found that falls were age-related and increased with age (see Table 2).

### 3.2. Comparison of Related Indicators of Elderly Patients in the Fall Group and the Nonfall Group

The elderly who fell or not within one year were surveyed and statistically processed. As shown in Table 3 below, there was no significant difference in height, age, and weight.

#### 3.2.1. Comparison of Basic Indicators

An independent sample *t*-test was performed on the data of the falling group and the nonfalling group. The results showed that the lean body mass *P* = 0.043, the gender *P* = 0.000, and the difference were statistically significant, and there was a significant difference between the groups, *P* = 0.44, on the MBI index, *P* > 0.05, which is not statistically significant, see Table 4.

#### 3.2.2. Comparison of Perceptual Functions

The observed sensory index data, using *t*-test and self-sampling, respectively, and statistical analysis, found that there is no obvious difference between the normal fall group and the normal fall group. Conclusion is as follows: the lower extremity activity sensation *P* < 0.05 is statistically significant compared with the control group, see Table 5.

#### 3.2.3. Comparison of Balance Ability

*(1) Standing on Both Feet-Eyes Open and Eyes Closed*. Legged stance index was calculated by single-case *t*-test. The analyzed data are shown in Table 6. When the eyes are closed, there is no significant difference in the indicators of falling and not falling; when the patient opens his eyes, the envelope length and the full length of the center of gravity pressure are significantly different. There was a significant difference between the patients who fell and those who did not fall. *P* < 0.05 for the envelope area and the horizontal swing of the pressure center of gravity is as follows, and there was a significant difference between the patients who fell and those who did not fall.

*(2) Standing on One Foot-Eyes Open and Eyes Closed*. The purpose of this test was to compare the balance of eyes open and closed on one foot between those who had fallen and those who had not fallen, and the results showed no significant difference between the two indicators, see Table 7.

#### 3.2.4. Univariate Analysis of Balanced Indicators

Taking the risk factors of falls in elderly patients as the main variable and whether or not falling was the main variable, the single linear regression method was used to explore various factors related to falls.

*(1) Univariate Analysis of Static Balance Index*. Standing on Both Feet-Eyes Open and Eyes Closed

When standing on two feet or with eyes open, a preliminary analysis of three factors related to falls, including envelope area, length of pressure center of gravity, and lateral sway of pressure center of gravity, was carried out, while when standing on two feet, no findings were found. Factors were associated with falls (Tables 8 and 9).

Standing on One Foot-Eyes Open and Eyes Closed

When standing on one foot, using the data of eyes open and closed as independent variables, and the fall accident as the dependent variable, multiple linear regression was performed, and no factors related to falls were found (Tables 10 and 11).

## 4. Screening of Fall Risk-Sensitive Indicators and Establishment of Models

According to the above results, the multifactor unconditional logistic regression was used for statistical test, the probability of inclusion was 0.05, whether the elderly fell as the dependent variable, the possibility of exclusion was 0.1, and the statistical method was carried out by gradual regression. The five indicators in the statistical sensitivity index, gender, posture sense of knee joint activity, capsule area at foot opening, length of pressure center, and lateral shaking of pressure center, are the main causes of falls in the elderly, as shown in Table 12.

ROC is a typical measurement method of specificity and sensitivity. ROC is a working characteristic, which determines its specificity and sensitivity according to a certain threshold point, and expresses the specificity and sensitivity in the form of graphics.  Figure 2 shows the ROC curve with 1-specificity on the abscissa and sensitivity on the ordinate, and the region consisting of the curve and the coordinate axis can be evaluated for the accuracy of the model. In the chart, from left to right, from left to right, and from left to right, as the area under the curve approaches 1, the prediction accuracy of the model is better, between 0.7 and 0.9, and the model is around 0.704, indicating that the pattern is correct.

After the goodness-of-fit test, *X*^2^ was 5.301, and *P* was 0.703, indicating that the formula can well explain the relationship between the five factors and the risk of falling. Therefore, the selection of the sensitivity index can well predict the risk of falling. Taking the fall accident as the benchmark, the samples of this pattern are grouped back and replaced, and the following data are obtained (see Table 13):

It can be concluded from the table that specificity = 8/13 = 61.54%, where sensitivity is 5/7 = 71.43%, and Error probability = 1 − specific = 38.46%.

It can be seen from the above results that the model has good specificity and sensitivity and has a small error prediction ability; so, the model is more reasonable.

## 5. Conclusion

In this study, through questionnaires, laboratory tests, and other methods, the correlation between different influencing factors and the risk of falling in the elderly was explored, the relevant factors were found out, and a corresponding prediction model was constructed accordingly, which is helpful for my country's entry into the aging society. Prevention work has laid a solid theoretical basis. From the above analysis, the following points are obtained:

1. The subjects in this paper are all 65 years old and the elderly. The survey data can be used as the basis for reducing falls in the elderly
2. The data statistics show that the selected predictors have a good forecasting effect, but there are differences in the scope of their influence, which can be used for targeted research
3. For the elderly who have fallen, the factors such as balance ability, active position sense function of the knee joint, eye opening envelope area, length of pressure center of gravity, and amplitude of lateral swaying of center of gravity are all risk factors for falling. The method has good accuracy and a good false positive rate and can be used for the effectiveness analysis of clinical treatment

## Figures and Tables

**Figure 1:** Fall time.

**Figure 2:** ROC curve.

**Table 1:** Subject's basic information.

Parameter	Minimum	Maximum	*X* ± *S*
Age	65.00	71.00	67.08 ± 2.19
Height (cm)	149.50	170.50	159.85 ± 6.59
Weight (kg)	41.20	76.05	63.68 ± 9.54
BMI	18.43	27.96	24.81 ± 2.54

**Table 2:** Gender and age distribution of fall events.

Age	Female_			Male_		
	*n*	*N* number	Fall rate	*n*	*N* number	Fall rate
65-70	7	4	57%	3	1	33%
71-75	5	3	60%	5	1	80%

**Table 3:** Subject's basic information.

Project indicators	Fall group	No fall group	*P*
Age	70 ± 3.79	68.38 ± 2.72	0.31_
Height (cm)	162.8 ± 5.33	161.11 ± 7.14	0.55_
Weight (kg)	64.28 ± 6.43	60.51 ± 12.25	0.90_

**Table 4:** Basic index comparison.

Project indicators	Fall group	No fall group	*P*
BMI	24.25 ± 2.10	23.20 ± 3.81	0.44_
Lean body mass (kg)	42.57 ± 6.00	50.90 ± 11.16	0.4_
Sex (male)	71.40 ± 3.91	67.33 ± 3.21	0.01
Gender (female)	69.00 ± 3.65	65.00 ± 2.55	0.01

**Table 5:** Perceptual metric comparison.

Project indicators	Fall group	No fall group	*P*
Vision	4.59 ± 0.14	4.61 ± 0.09	0.73
Active position sense (°)	5.34 ± 1.31	6.78 ± 1.66	0.04
Passive position sense (°)	6.23 ± 1.65	5.68 ± 1.11	0.743

**Table 6:** Comparison of eye-opening and eye-closing indicators when standing on both feet.

Project indicators	Feet-eyes open			Feet-eyes closed		
	Fall group	No fall group	*P*	Fall group	No fall group	*P*
Envelope length (mm)	17.43 ± 3.32	13.47 ± 1.87	0.007	17.10 ± 4.03	14.42 ± 2.04	0.102
Envelope area (mm^2^)	170.28 ± 27.85	138.83 ± 39.08	0.049	166.94 ± 27.90	138.83 ± 39.08	0.076
Envelope angle (°)	59.50 ± 15.33	44.60 ± 23.67	0.103	47.84 ± 14.29	42.10 ± 25.08	0.521
Overall length of pressure center of gravity (mm)	303.85 ± 41.49	233.74 ± 43.64	0.002	287.19 ± 46.19	258.74 ± 20.38	0.121
Horizontal swing of pressure center of gravity (mm)	2.48 ± 0.99	3.42 ± 0.67	0.031	3.06 ± 0.87	3.42 ± 0.67	0.338
Pressure center of gravity vertical swing (mm)	4.07 ± 0.57	4.41 ± 0.30	0.142	4.40 ± 0.74	4.91 ± 0.48	0.107
Percentage of pressure on right foot (%)	46.19 ± 5.85	45.36 ± 3.47	0.725	46.52 ± 6.17	45.36 ± 3.47	0.637
Percentage of pressure on left foot (%)	51.06 ± 6.40	50.14 ± 5.00	0.738	51.06 ± 6.40	50.64 ± 4.78	0.878

**Table 7:** Comparison of eye-opening and eye-closing indicators when standing on one foot.

Project indicators	Feet-eyes open			Feet-eyes closed		
	Fall group	No fall group	*P*	Fall group	No fall group	*P*
Envelope length (mm)	18.02 ± 3.08	15.73 ± 2.02	0.082	19.68 ± 3.45	18.60 ± 1.89	0.432
Envelope area (mm^2^)	175.28 ± 25.92	163.83 ± 48.26	0.498	188.83 ± 25.80	179.44 ± 22.77	0.403
Envelope angle (°)	64.84 ± 12.91	50.85 ± 18.45	0.061	69.84 ± 14.27	59.60 ± 11.23	0.106
Overall length of pressure center of gravity (mm)	336.35 ± 36.03	311.24 ± 34.39	0.138	361.35 ± 49.99	336.24 ± 42.90	0.261
Horizontal swing of pressure center of gravity (mm)	3.06 ± 0.83	3.67 ± 0.31	0.065	3.56 ± 1.00	4.42 ± 1.01	0.078
Pressure center of gravity vertical swing (mm)	4.32 ± 0.46	4.66 ± 0.50	0.137	4.57 ± 0.44	5.04 ± 0.74	0.094
Percentage of pressure on right foot (%)	47.02 ± 7.01	50.24 ± 6.17	0.307	48.69 ± 6.28	52.74 ± 5.70	0.161
Percentage of pressure on left foot (%)	52.39 ± 6.50	57.02 ± 6.02	0.126	56.97 ± 8.41	63.89 ± 6.61	0.067

**Table 8:** Univariate logistic regression analysis of standing with eyes open.

Project indicators	Regression coefficients	Standard error	*P*
Envelope length (mm)	-0.792	0.407	0.009
Envelope area (mm^2^)	0.061	0.098	0.047
Envelope angle (°)	0.816	0.295	0.093
Overall length of pressure center of gravity (mm)	0.009	0.009	0.004
Pressure center of gravity horizontal swing (mm)	0.658	0.029	0.031
Pressure center of gravity vertical swing (mm)	2.315	0.741	0.128
Percentage of pressure on right foot (%)	0.141	0.173	0.707
Percentage of pressure on left foot (%)	0.027	0.680	0.870

**Table 9:** Univariate logistic regression analysis of standing with eyes closed.

Project indicators	Regression coefficients	Standard error	*P*
Envelope length (mm)	-0.005	-0.005	0.999
Envelope area (mm^2^)	0.006	0.006	0.511
Envelope angle (°)	0.001	0.025	0.218
Overall length of pressure center of gravity (mm)	-0.017	0.028	0.505
Pressure center of gravity horizontal swing (mm)	0.001	0.004	0.852
Pressure center of gravity vertical swing (mm)	-0.002	0.006	0.773
Percentage of pressure on right foot (%)	-0.030	0.089	0.801
Percentage of pressure on left foot (%)	0.031	0.091	0.702

**Table 10:** Univariate logistic regression analysis of standing on one foot with eyes open.

Project indicators	Regression coefficients	Standard error	*P*
Envelope length (mm)	-0.001	0.001	0.509
Envelope area (mm^2^)	0.000	0.002	0.421
Envelope angle (°)	0.002	0.005	0.408
Overall length of pressure center of gravity (mm)	0.007	0.018	0.545
Pressure center of gravity horizontal swing (mm)	0.005	0.011	0.531
Pressure center of gravity vertical swing (mm)	-0.001	0.003	0.796
Percentage of pressure on right foot (%)	-0.080	0.080	0.308
Percentage of pressure on left foot (%)	0.071	0.076	0.902

**Table 11:** Univariate logistic regression analysis of standing on one foot with eyes closed.

Project indicators	Regression coefficients	Standard error	*P*
Envelope length (mm)	0.001	0.001	0.845
Envelope area (mm^2^)	0.001	0.001	0.407
Envelope angle (°)	0.001	0.003	0.959
Overall length of pressure center of gravity (mm)	0.005	0.001	0.984
Pressure center of gravity horizontal swing (mm)	-0.006	0.010	0.425
Pressure center of gravity vertical swing (mm)	-0.006	0.005	0.648
Percentage of pressure on right foot (%)	0.079	0.065	0.102
Percentage of pressure on left foot (%)	-0.039	0.065	0.100

**Table 12:** Unconditional logistic regression analysis of risk factors for falls.

Project indicators	Regression coefficients	Standard error	*P*
Constant	-12.904	4.279	0.004
Gender	0.905	0.239	0.001
Active position sense of the knee joint (°)	0.034	0.021	0.043
Eye opening envelope area of both feet (mm^2^)	0.001	0.000	0.047
Full length of center of gravity with both feet open and eyes open (mm)	0.005	0.001	0.045
Pressure center of gravity swing horizontally with both feet open (mm)	.235	0.091	0.002

**Table 13:** Results of 3 back substitutions.

Whether there is a history of falls			
Model judgment	Yes	No	Total
Yes	5	5	1 0
No	2	8	1 0
Total	7	1 3	2 0

## Data Availability

The dataset used in this paper are available from the corresponding author upon request.
